The article "Evaluation of Airborne Asbestos Concentrations Associated with the Operation and Maintenance of Brakes and Clutches on Nonautomated Heavy Equipment" was published in 2022. Journal: J Environ Public Health.

# Evaluation of Airborne Asbestos Concentrations Associated with the Operation and Maintenance of Brakes and Clutches on Nonautomated Heavy Equipment

**DOI:** 10.1155/2022/9831883

**Published:** 2022-04-22

**Authors:** J. Sahmel, H. Avens, T. Ferracini, A. Banducci, K. Rickabaugh

**Affiliations:** ^1^Insight Exposure and Risk Sciences, 1790 38^th^ Street, Suite 201, Boulder, CO 80301, USA; ^2^RJ Lee Group, 350 Hochberg Rd, Monroeville, PA 15146, USA

## Abstract

This study evaluated the potential for chrysotile asbestos exposure during maintenance and operation of older, nonautomated heavy equipment with chrysotile-containing brake and clutch linings. Recent reports indicate that such equipment may be in current use in the U.S. and other locations, including developing countries, due to its lower cost and ease of maintenance compared to newer equipment. Personal and area airborne fiber concentrations were measured for cranes with draglines during brake and clutch repair, equipment operation, shop cleanup, and clothes handling of the mechanic's coveralls over a period of three days. The range of airborne chrysotile concentrations during the complete friction band replacement process, including band removal from the equipment, friction lining replacement, and reinstallation, ranged from 0.0053 to 0.0273 f/cc (phase contrast microscopy-equivalent or PCME) over 3.3 to 6.2 hours. Additional bench work tasks, including electric wire brushing, hand sanding, riveting, and compressed air use were also performed. Full shift airborne chrysotile concentrations (6.1–8.5 hours) for all combined maintenance activities were 0.0093, 0.0414, and 0.0445 f/cc (PCME), on days 1, 2, and 3, respectively. Personal short-term samples (14–36 minutes) for lining removal, installation, wire brushing, hand sanding, and compressed air use ranged from nondetect (ND) to 0.238 f/cc (PCME), below the U.S. Occupational Safety and Health Administration's (OSHA's) 30-minute excursion limit of 1 f/cc. Short-term samples during crane operation, shop cleanup, and simulated laundry activities with the mechanic's coveralls ranged from ND to 0.01 f/cc (PCME; 15–36 minutes). The results indicated that full-shift measured airborne chrysotile concentrations during the brake and clutch maintenance activities evaluated remained below the U.S. 8-hour time-weighted average (TWA) permissible exposure limit (PEL) for asbestos of 0.1 f/cc. The results are likely to be relevant to farmers, construction workers, and vehicle maintenance workers historically, as well as today for those who choose to continue using and maintaining such equipment.

## 1. Introduction

The design of friction wear products such as brake or clutch linings must consider important safety factors including wear, stability, and the ratio of brake torque to applied force [1]. Historically, such linings contained chrysotile asbestos due to its unique properties, including strength, resistance to heat, and binder properties [2]. Certain brake linings and pads historically contained approximately 30% to 70% chrysotile by weight before use [3–6]. Similarly, certain clutch discs or components were historically comprised of approximately 20 to 55% chrysotile [7–11].

Chrysotile is one of six asbestos mineral fiber types identified by the Occupational Safety and Health Administration (OSHA) in the U.S. [12]. Chrysotile is a hydrated magnesium silicate in the serpentine mineral class that forms soft and flexible fibers, whereas the other primary class of asbestos minerals identified by OSHA, the amphiboles (such as crocidolite or amosite), generally contains iron and forms rigid fibers [13, 14]. Over a number of decades, evidence has accumulated in the published literature demonstrating that there are significant differences in cancer potency according to the different mineral fiber types, with chrysotile being the least potent of the common industrial fiber types for both lung cancer and mesothelioma induction (if chrysotile is capable of inducing mesothelioma at all), and crocidolite typically being the most potent of the mineral fiber types that have been used commercially [15–20]. Chrysotile has been reported to be ubiquitous in the background or ambient environment [21]. Measurements of ambient asbestos concentrations in recent decades have ranged from nondetectable to 0.0047 f/cc (outdoors) and nondetectable to 0.012 f/cc (indoors) for fibers at least 5 *μ*m in length in long-term samples of up to approximately 13 hours or more [22, 23].

A number of peer-reviewed and government studies have been published since the 1970s that have reported the long-term or full-shift airborne fiber concentrations associated with the work of automotive and equipment mechanics performing a variety of tasks related to chrysotile-containing brakes and clutches [9, 10, 24–42]. Along with analyses from OSHA, the National Institute for Occupational Safety and Health (NIOSH), and the U.S. Environmental Protection Agency (U.S. EPA), these studies collectively indicate that the potential for chrysotile exposure during the maintenance of asbestos-containing brakes and clutches is below the current occupational full-shift 8-hour time-weighted average (TWA) permissible exposure limit (PEL) for asbestos in the U.S. of 0.1 f/cc [30, 43, 44]. These analyses are also consistent with studies that have evaluated the cumulative exposure potential associated with automotive mechanic work over time [45, 46].

Nearly all of these studies, however, evaluated the potential for asbestos exposure associated with passenger vehicles, trucks, or buses. Few studies have evaluated the potential for exposure during work with or around heavy equipment, which compared to passenger vehicles, trucks, and buses, may have unique designs and uses. Specifically, the current study evaluated potential exposures from chrysotile-containing brakes and clutches during operation and maintenance of nonautomated cranes with draglines manufactured in the 1950s and 1960s. Such equipment has been used for a variety of applications including earth moving, highway construction, and mining. Furthermore, recent news reports in the U.S. have pointed to the increasing use of nonautomated heavy equipment that is 40 years old or older because of its less complicated machinery, ease of repair in the field, and lower costs associated with maintenance and repair [47, 48]. Therefore, characterization of potential chrysotile exposures associated with operation and repair of this nonautomated heavy equipment remains relevant today, not only in the U.S. but also in developing countries where farmers, construction workers, and small business owners may still be routinely using such equipment.

There are some challenges to interpreting some of the previously published airborne fiber concentration data associated with brake and clutch work. First, some older studies reported measurements based only on phase-contract microscopy (PCM), which is not specific to asbestos fibers [4, 24, 49]. PCM is a straightforward and cost-effective method that counts all fibers meeting the size criteria of at least 5 *µ*m in length and 0.25 *μ*m in width with a 3 : 1 aspect ratio, regardless of whether the fibers are asbestos or not [50]. Due to pressure and heat generated during the braking process, an extremely large fraction of the fibers in the friction wear debris are reported to be nonasbestos, such as forsterite, a degradation product of chrysotile [10, 41, 51–55]. The PCM method will still count these nonasbestos fibers, which could lead to an overestimate of asbestos exposure potential [30, 45, 52, 53, 56, 57].

Second, some studies have measured airborne asbestos concentrations using transmission electron microscopy (TEM) [26–29, 52]. Unlike PCM, TEM can distinguish between asbestos and nonasbestos fibers [58]. TEM can also identify fibers as short as 0.5 *μ*m in length and <0.1 *μ*m in width; however, OSHA and the U.S. EPA specify that asbestos fibers ≥5 *μ*m in length with at least a 3 : 1 aspect ratio are the appropriate dimensions to use for asbestos exposure and risk assessment [58–62]. The vast majority of airborne asbestos fibers associated with brake and clutch maintenance as measured by TEM are reportedly much shorter than 5 *μ*m in length [45, 51, 52, 63, 64]. The TEM method alone may therefore report concentrations that are higher or far higher than the concentrations applicable to U.S. regulatory risk assessment. The best metric for exposure assessment of brake and clutch work is, therefore, the PCM-equivalent or PCME concentration, which is calculated by multiplying the PCM fiber concentration by the percent of fibers that are specifically asbestos, as measured by TEM (as specified by NIOSH method 7402) [50, 65, 66].

Third, previous studies that have measured airborne fiber concentrations associated with brake or clutch maintenance work have reported a wide range of sampling durations, many of which were not long-term or full-shift, or in some instances, a sampling duration was not reported at all [4, 45, 52, 55, 63, 67, 68]. Sampling for less than a full work shift (typically 8 hours) precludes direct comparison against important benchmarks such as the OSHA 8-hour TWA PEL without additional consideration of exposure potential during the time outside of the recorded sample duration. For example, peak exposures over a several-minute period are not directly comparable or relevant to a worker's exposure potential over the full task or workday [45, 69]. The omission of sampling duration, or the use of partial-shift or peak sampling duration alone, limits the ability to interpret airborne fiber concentration measurements with respect to occupational exposure standards or other risk assessment benchmarks [70, 71]. While task-based exposures can be valuable to characterize specific activities, they are most helpful when considered in the context of full-shift measurements.

Only two published studies were identified that evaluated airborne chrysotile concentrations associated with work on heavy equipment brakes or clutches, one of which evaluated brake and clutch replacements [41], and another which collected short-term measurements during brake removal [55]. Neither study evaluated chrysotile exposure potential from maintenance work on cranes. Additionally, a single unpublished study was identified that evaluated the potential for chrysotile exposures during the operation of heavy equipment [72]. Collectively, while informative, these studies do not address the full range of activities that may be performed by heavy equipment brake or clutch mechanics and operators. Additional study is therefore warranted to better characterize the potential for chrysotile exposures associated with the range of maintenance activities and operational scenarios that may be encountered with chrysotile-containing brakes and clutches on heavy equipment.

To address the data gaps, the current study measured airborne chrysotile concentrations during the full workday and for specific short-term tasks associated with the maintenance and operation of nonautomated crane equipment. The assessment included a variety of friction lining manipulation tasks that heavy equipment mechanics may perform, including tasks not previously evaluated in the peer-reviewed literature. For example, separate task-based samples were collected during electric wire brush cleaning of heavy equipment friction linings, during hand sanding of linings, and during the isolated compressed air blow-off of linings. Additionally, the cranes evaluated had brakes and clutches that were open to the air and adjacent to the equipment operator (Figure 1), a configuration not previously evaluated for operator exposure potential. The full-shift measurements collected during this study also covered the duration of all brake and clutch maintenance activities that were evaluated, enabling direct comparison to the OSHA 8-hour TWA PEL. Both the PCM and TEM (PCME) methods were used, facilitating comparisons between asbestos and nonasbestos airborne fiber concentrations. Overall, this study contains a number of measurements that add substantially to the relatively limited body of research related to chrysotile exposure potential during heavy equipment repair and operation. While these data are relevant for understanding the historic potential for asbestos exposure during the use of such equipment, the results remain relevant today due to the continued use of some older, nonautomated heavy equipment that can have greater simplicity of use and lower cost of repair compared to newer models.

## 2. Methods

Brake and clutch work on heavy equipment was performed in a commercial repair and maintenance garage located outside of Lancaster, Pennsylvania, from January 5 to 7, 2021. IRB approval was obtained for the protocol prior to the study (WCG IRB Study Number 1298632). Additionally, a COVID-19 protocol was in place that required all individuals on-site to wear an N95 disposable respirator (at a minimum), if not a more protective respirator, for the entire duration of the study. All air and bulk samples in this study were collected and analyzed using generally accepted standard methods, and citations have been provided to all relevant method numbers and dates. Samples were obtained under the direct supervision of a certified industrial hygienist (CIH) and sample analyses were conducted by a laboratory accredited (ref. ISO 17025 : 2017) to perform asbestos analysis.

Maintenance work was performed on a Bucyrus-Erie 22B crane manufactured in 1953 (Milwaukee, Wisconsin, USA; serial number 105960) and a Bucyrus-Erie 15B crane manufactured in 1960 (Milwaukee, Wisconsin, USA; serial number 121137). The work was performed by a career mechanic with over 36 years of experience working with heavy equipment, including cranes. The approximate garage dimensions were 48.8 m by 21.3 m with a 7.9 m ceiling (Figure 2). The garage was enclosed and had no mechanical ventilation. The study also evaluated the operation of a Bucyrus-Erie 22B crane (Milwaukee, Wisconsin, USA; serial number 126638) with a dragline outside of the garage by a heavy equipment operator with over 30 years of experience operating this type of equipment. Figures 1(a), 1(b), and 1(e) depict the 22B crane used for the operation assessment, and this crane was similar to the 22B and 15B cranes used for the maintenance activities.

### 2.1. Bulk Sampling

All friction linings removed, installed, manipulated, or used in the study were sampled in advance for asbestos content. Multiple sets of original, unused, predrilled Bucyrus-Erie replacement clutch and brake linings that were designed for use with the crane equipment evaluated were available and used in the study. The linings consisted mostly of dark brown or dark gray composite material manufactured by American Brakeblok (Detroit, Michigan, USA) (Figure 1(h)). Where noted, light gray woven friction lining material (unknown supplier) was also bulk tested and used in the study. A total of 18 bulk samples from clutch lining material and 19 bulk samples from brake lining material were collected from both the new and used linings. Asbestos content was determined by polarized light microscopy (PLM) using the quantitative point count methodology (EPA Method 600/R-93/116). Samples were subjected to gravimetric reduction by ashing and acid treatment methods prior to PLM analysis. The bulk asbestos concentrations were calculated and reported on a total amount per sample basis. Bulk sampling of the brake and clutch linings already on the cranes did not require disassembly because the assemblies were not enclosed.

### 2.2. Air Sampling

Air samples were collected during maintenance, operation, and clothes handling activities. Samples were collected and analyzed using the PCM method (NIOSH Method 7400). A TEM (NIOSH Method 7402) analysis was also performed if a detectable PCM concentration was reported. The combined results of the PCM and TEM samples were used to calculate PCME concentrations where applicable, according to NIOSH Method 7402. All air samples were collected using 25 mm diameter, 0.8-micron pore size mixed cellulose ester (MCE) membrane filters preloaded in carbon-filled black polypropylene conductive cassettes with 50 mm extension cowls (SKC, Eighty-Four, Pennsylvania, USA). Air samples were collected with SKC AirCheck TOUCH personal pumps (Eighty-Four, Pennsylvania, USA) and Allegro Industries Rotary Vane stationary pumps (Piedmont, South Carolina, USA). The flow rate was calibrated before and after sample collection with a Bios Defender 510M or 510H calibrator (Butler, New Jersey, USA). Two baseline area air samples were collected at the beginning of the study to test for any preexisting detectable airborne fibers in the workplace (30-minute duration, ∼10 L/min flow rate). Throughout the study, outdoor background area air samples were also collected to evaluate airborne fiber concentrations at the study location (partial/full-shift duration, ∼5 L/min flow rate).

To evaluate particle characteristics, three additional air samples were collected using 25 mm diameter, 0.4-micron pore size polycarbonate (PC) filters (SKC, Eighty-Four, Pennsylvania, USA) preloaded in carbon-filled black polypropylene conductive cassettes with 50 mm extension cowls. The PC filters obtained were analyzed and imaged using scanning electron microscopy (SEM) techniques. The samples for SEM analysis were collected during two compressed air blowout tasks and a woven lining installation task.

#### 2.2.1. Mechanic Work

Over a three-day study period, mechanic personal breathing zone and area (bystander and ambient) samples were collected during the removal and replacement of brake and clutch bands on the two cranes (Figure 3). The mechanic was asked to perform maintenance activities on the 22B crane on days 1 and 2 and on the 15B crane on day 3 using his standard work practices. This work included removing a brake or clutch band from a crane, bringing the metal band to a workbench, removing and replacing the lining, and then reinstalling the band into the crane. This series of tasks is referred to as “Crane Maintenance.” On days 2 and 3, the mechanic was asked to perform additional tasks of interest at the workbench on 22B and 15B brake and clutch bands and linings which had already been removed from the crane equipment before the study started. These tasks are referred to as “Additional Maintenance Tasks.” Some of these additional tasks were not part of the mechanic's standard work practices but were selected based on work practices described in previous literature and the potential to generate dust.

Full-shift, partial-shift, and task-based personal samples were collected from the mechanic's breathing zone during clutch and brake work. Task-based area samples were also collected 1.5 m from the workbench. Full-shift area samples were collected at 1.5 m and 4.6 m from work performed on the 22B and 15B cranes, as well as 4.6 m from the workbench. Full-shift ambient (remote area) samples were collected 9.1 m from the work at the crane and 9.6 m from the workbench. Sampling flow rates of approximately 1-2 L/min were used for personal sampling, while approximately 5 L/min was used for area samples. Sampling locations are depicted in Figure 2.  Table 1 provides an overview of the air samples collected.

#### 2.2.2. Crane Maintenance

The mechanic removed, relined, and reinstalled a clutch band and a brake band from the 22B crane, removed a clutch band and brake band from the 15B crane, and relined the 15B clutch band (Figure 3). The metal bands (clutch and brake) were circular in shape to fit around the associated drum and were not enclosed in any housing. The clutch linings were attached to the outside perimeter of the metal clutch band (Figure 1(d)), whereas the brake linings were attached to the inside perimeter of the metal brake band (Figure 1(c)).

The mechanic removed the brake and clutch bands from the cranes using hand tools, a pneumatic impact wrench, spray lubricant, and a torch as needed. He then brought the metal clutch or brake bands to a workbench to remove the clutch or brake linings from the metal bands. The mechanic used an electric grinder as needed to remove the heads of rivets attaching the linings to the band. A hammer and punch were subsequently used to remove the remaining portion of the rivet, allowing the linings to be detached from the metal band.

Prior to attaching replacement linings at the workbench, rust and debris were removed from the metal band either by a pneumatic sander (SM P-80 grit sandpaper) or an electric wire brush. The metal band was then blown off with compressed air, painted, and allowed to dry for a minimum of 15 minutes. The mechanic then attached the new linings to the metal band by inserting rivets into the factory-predrilled holes. The metal clutch and brake bands with new linings were subsequently reinstalled on the crane.

#### 2.2.3. Additional Maintenance Tasks

In addition to brake and clutch band removal, relining, and reinstallation in the cranes, the mechanic also performed specific additional short-term maintenance tasks of interest using clutch and brake linings and bands that were removed from cranes before the study started. Specifically, six additional clutch and brake maintenance activities were performed by the mechanic at the workbench (Figure 3). The first and second tasks involved compressed air blowoff of used 15B and 22B brake linings and used 15B and 22B clutch linings, respectively. The third task comprised hand sanding of used 22B brake linings followed by debris removal with compressed air. In the fourth task, the mechanic removed 22B brake linings and then cleaned and painted the metal bands following the removal of the linings. The fifth task included cleaning the surface of used 22B brake linings with an electric wire brush, and the sixth event involved the attachment of a new woven brake lining material to a brake band. To install the woven lining, the mechanic cut the lining to length with a hacksaw, used a pneumatic drill to create rivet holes in the woven lining, countersunk the rivet holes on the opposite side of the lining, removed debris from the rivet holes with compressed air, and installed the rivets. Figure 1 depicts many of the tasks that were performed at the workbench.

#### 2.2.4. Shop Cleanup

At the end of each day, the mechanic spent two to three minutes manually sweeping the debris generated from the daily brake and clutch work activities with a broom and brush, including the floor and tarps covering the floor near and around the 22B and 15B cranes and at the workbench. Regarding general cleanup, the mechanic explained that, to prevent dust and debris from settling in the bearings and grease on the crane, compressed air was never used inside the cab or on the crane itself for cleaning or any other purpose.

#### 2.2.5. Crane Operation

Personal and area air samples were collected during 30 minutes of outdoor crane operation (∼4 L/min flow rate). Stationary area air samples were collected at 2.4 m and 2.9 m from the sides of the crane cab at a height of approximately 1.4 m. The side of the crane where the operator entered the cab and the side panel on the opposite side of the cab were open during sampling. Prior to sampling, the crane was started to warm up the levers, boom, and shovel for approximately 30 minutes. Sampling began while the crane was idle; within five minutes, the operator started operating the shovel continuously to scoop and move dirt using the dragline until the end of the 30-minute sampling period. Operation of the crane consisted of (1) swiveling the cab left and right, (2) lowering and raising the shovel, and (3) scooping and releasing the shovel via the hoist. The crane boom was fixed and did not independently move during the study.

#### 2.2.6. Clothes Handling/Laundering

On day 3 of the study, a clothes laundering simulation was conducted which consisted of handling the three sets of new coveralls that were worn by the mechanic during brake and clutch work (one for each day of the study). Personal samples were collected during a 15-minute clothes handling period during which the subject shook out each coverall, checked pockets, turned the coveralls inside out and right side in, placed them in a pile, and repeated these steps for 13 minutes. The final two minutes of sampling consisted of sweeping the floor underneath the clothes handling area with a broom and dustpan. Following clothes handling, two stationary samples were subsequently collected immediately afterwards for a 15-minute dust settling period. All samples were collected at approximately a 10 L/min flow rate.

### 2.3. Statistical and Data Analysis Methods

Statistical and data analyses were conducted using MS Excel (Office 2019; Microsoft; Redmond, Washington, USA). U.S. EPA guidance regarding airborne samples states that “when computing the mean of a set of asbestos measurements, samples that are “non-detect” should be evaluated using a value of zero,” explaining that “use of 1/2 the sensitivity as a surrogate for asbestos non-detects may lead to a substantial overestimate of the true mean of a group of samples” [60]. Following U.S. EPA guidance, samples which were below the analytical sensitivity limit and considered nondetectable (ND) by PCM were treated as zero values when calculating average concentrations for both PCM and PCME. For samples that were above the PCM analytical sensitivity limit but had no detected asbestos fibers by TEM, the PCM fiber concentration was used when calculating PCM averages, while zero was used when calculating the PCME average [60].

## 3. Results

During the study, ambient temperatures inside the garage ranged from 6.7 to 7.2°C (44.1-45°F), with relative humidity between 58 and 68%. During crane operation, the outdoor temperature was 3.3 to 3.9°C (38–39°F), the relative humidity was 54 to 59%, and the reported wind speed at the nearby Lancaster Airport was approximately 19 kph (12 mph) NW.

### 3.1. Bulk Sampling

All of the brake and clutch lining materials tested contained chrysotile asbestos ranging in content from 22 to 41%. In addition, the woven brake lining material that was installed on a 22B brake band on day 3 contained 31 to 35% chrysotile. Furthermore, one bulk sample of dust was collected from the surface of the mechanic's workbench following the removal of clutch band linings and rivets on day 1 of the study. This sample consisted primarily of metal particulates, and no asbestos fibers were detected. No amphibole fibers were detected in any of the bulk lining materials tested.

### 3.2. Air Sampling

Personal and area samples were collected during brake and clutch maintenance work, crane operation, and clothes handling following maintenance work. Measured full-shift and half-shift airborne fiber concentrations are presented in Table 2, and task-based airborne fiber concentrations are presented in Table 3. TEM analyses were conducted for all samples with fibers above the PCM sensitivity limit. No asbestos fibers were identified by PCM and/or TEM in any of the blank samples, and no amphibole fibers were detected in any of the air samples. Baseline area air samples collected at the start of the study had no detected airborne fibers (<0.009 f/cc, *N* = 2). The average full-shift outdoor concentration across all three days was 0.00047 f/cc (PCME), including two days for which no fibers were detected and one day with a TWA chrysotile concentration of 0.0014 f/cc (PCME) (Table 2).

#### 3.2.1. Clutch and Brake Work

*(1) Personal Samples*. One full-shift sample was collected each day on the mechanic's left lapel. A set of half-shift samples was also collected each day on the mechanic's right lapel, and these were averaged to provide a second evaluation of the full-shift airborne concentration. The measured and calculated full-shift personal airborne concentrations were also averaged for each day, yielding 0.0168, 0.0414, and 0.0499 f/cc (PCM) for days 1–3, respectively, and an overall average of 0.0344 f/cc (PCM) across all three days (Table 2). The associated chrysotile-specific fiber concentrations were 0.0093, 0.0414, and 0.0445 f/cc (PCME), with an overall average of 0.0317 f/cc (PCME). All measured and calculated full-shift concentrations were below OSHA's 8-hour TWA PEL of 0.1 f/cc.

A description of the tasks performed by the mechanic each day and the associated fiber concentrations are shown in Table 3. A summary of all events performed over each day is depicted in Figure 3. As previously noted, some tasks were part of a complete or partial brake or clutch replacement conducted by the mechanic following his typical work practices (“Crane Maintenance” in Figure 3), while other tasks involved manipulation of linings that were removed from cranes before the study started (“Additional Maintenance Tasks”).

TWA chrysotile concentrations specifically during Crane Maintenance activities were 0.0053, 0.0132, and 0.0143 f/cc PCME on day 1 based on the full-shift, partial-shift, and task-based samples, respectively, (6.2, 6.1, and 5.8 hours); 0.0273 f/cc PCME on day 2 based on the 1^st^ six task-based samples collected that day (6.1 hours); and 0.0215 and 0.0196 f/cc PCME on day 3 based on the 2^nd^ partial-shift, and the 5^th^, 6^th^, and 7^th^ task-based samples, respectively, collected that day (3.7 and 3.3 hours), for an overall range of 0.0053 to 0.0273 f/cc (PCME).

Task-based personal samples were collected on the mechanic's right lapel. Personal samples with sampling durations of approximately 30 minutes or less (14–36 minutes) ranged from ND to 0.238 f/cc (PCM and PCME) and were well below OSHA's 30-minute excursion limit of 1 f/cc (Table 3 and Figure 4). These tasks included removal, installation, electric wire brushing, hand sanding, compressed air blow-off of linings at the workbench, and cleanup. Short-term airborne fiber concentrations for the Additional Maintenance Tasks performed at the bench included 0.141 f/cc (PCME, 29 minutes) and 0.186 f/cc (PCME, 31 minutes) for greater than two minutes of compressed air use on old brake and clutch linings; 0.238 f/cc (PCME, 32 minutes) for approximately four minutes of hand sanding of brake linings followed by approximately one minute of compressed air use; and 0.189 f/cc (PCME, 30 minutes) for approximately two minutes of electric wire brush cleaning of brake linings. No chrysotile fibers were seen in the personal cleanup samples on days 1 and 2. One chrysotile fiber was observed in the personal cleanup sample on day 3; however, the sampling pump shut off prior to the completion of the sampling period, so the concentration is uncertain and is not presented in Table 3.

Personal samples collected for 38 to 60 minutes during bench work tasks included removal and installation of linings during clutch work (ND-0.077 f/cc PCM or ND-0.039 f/cc PCME) and installation of woven linings (60 minutes, 0.260 f/cc PCM and PCME). Longer duration personal task-based samples (72–200 minutes) collected during the installation and removal of clutch and brake bands from the cranes yielded concentrations ranging from ND to 0.050 f/cc by PCM (ND-0.044 f/cc by PCME).

*(2) Area Samples*. Full-shift area samples collected at 1.5, 4.6, and 9.1 m from the crane under repair were similar across each location, with 3-day average concentrations of 0.0029, 0.0026, and 0.0028 f/cc by PCM (0.0023, 0.0024, and 0.0025 f/cc by PCME), with increasing distance (Table 2). Likewise, full-shift area samples collected at 4.6 and 9.6 m from the workbench were similar, with 3-day averages of 0.0030 and 0.0033 f/cc by PCM (0.0024 and 0.0029 f/cc by PCME), respectively. These values were indistinguishable from the baseline area air measurements (<0.009 f/cc by PCME).

Task-based area samples were collected at a location that was approximately 1.5, 18, and 21 m from the workbench, 15B crane, and 22B crane. Task-based area samples (11- to 129-minute sampling durations) collected during Crane Maintenance and Additional Maintenance Tasks had concentrations ranging from ND to 0.087 f/cc (PCM) (up to 0.085 f/cc by PCME) (Table 3). Among these samples, matched personal and 1.5 m area samples (14 pairs) were available for all tasks conducted at the workbench.

*(3) Personal vs. Area Task-Based Samples*. Of the 14 pairs of matched measurements during bench work, the personal and area task-based samples had 5 and 9 ND samples by PCM, respectively. For the 9 personal samples above the PCM analytical sensitivity limit, their matched area fiber concentrations (PCM) were ND in four cases and were approximately 10 to 60% of the corresponding personal concentration in the remaining five cases. Similar results were seen for the PCME values. Regarding cleanup, two task-based samples that were collected 1.5 m from the workbench yielded <0.017 f/cc (PCM) and 0.051 f/cc (PCM and PCME), whereas personal cleanup concentrations were <0.045 and 0.059 f/cc (PCM) with no chrysotile fibers detected (PCME). Those samples with a duration of approximately 30 minutes or less during mechanic work were all below the OSHA 30 minute excursion limit of 1 f/cc (Figure 5).

#### 3.2.2. Crane Operation

Concentrations of <0.020 and 0.021 f/cc (PCM) were measured on the operator's right and left lapels during 30 minutes of crane operation (Table 3). TEM analysis of the PCM-detect sample identified one chrysotile and one nonasbestos fiber, resulting in a chrysotile concentration of 0.010 f/cc (PCME) and an average chrysotile concentration of 0.005 f/cc (PCME). No fibers were detected at 2.4 or 2.9 m on either side of the crane during operation.

#### 3.2.3. Clothes Handling

The handling and shakeout of the mechanic's three sets of coveralls and subsequent sweeping of the clothes handling area yielded 15-minute TWA concentrations of 0.095 and 0.079 f/cc (PCM), as measured on the left and right lapels of the clothes handler (Table 3). Based on TEM analysis, 6% or fewer of the fibers were chrysotile, yielding chrysotile concentrations of ND and 0.0044 f/cc (PCME), and an average chrysotile concentration of 0.0022 f/cc for the clothes handler. No fibers were detected in the clothes handling area during the 15 minutes immediately after clothes handling, yielding an average exposure of 0.0011 for the 30-minute period evaluated. Assuming no exposure for the clothes handler during the remainder of the workday, the calculated 8-hour TWA for clothes handling was 0.000069 f/cc (PCME), which was approximately 0.2% of the average full-shift mechanic exposure (0.0317 f/cc, PCME).

#### 3.2.4. SEM Analysis

SEM analysis demonstrated that some of the airborne particles collected during the study contained both fibers and other binder/debris material (Figure 6).

## 4. Discussion

This study assessed the potential for chrysotile exposure associated with the operation and maintenance of nonautomated cranes that employed asbestos-containing friction linings in brakes and clutches. As noted, all maintenance activities were performed in an enclosed garage with no mechanical ventilation, conditions expected to yield upper-bound airborne fiber concentrations due to limited airflow. Based on the results of the study, full-shift PCM and PCME airborne fiber concentrations for all activities evaluated were below the current OSHA 8-hour TWA PEL for asbestos of 0.1 f/cc and at times below the LOD. The full-shift airborne chrysotile concentrations over the three days of the study were 0.0093, 0.0414, and 0.0445 f/cc (PCME), respectively, over 6.1 to 8.5 hours, with an overall average of 0.0317 f/cc (PCME). A subset of the samples specifically evaluated airborne chrysotile concentrations during the routine flow and duration of typical crane maintenance work, excluding the additional maintenance tasks. These results, ranging from 0.0053 to 0.0273 f/cc (PCME) over 3.3 to 6.2 hours, are the most representative of brake and clutch maintenance work on this type of equipment. Despite the repeated additional bench work tasks performed on days 2 and 3, full-shift airborne chrysotile concentrations remained below the current OSHA 8-hour PEL on those days. These results are consistent with the conclusions of OSHA, NIOSH, and the U.S. EPA regarding full-shift airborne fiber concentrations associated with automotive mechanic work, which collectively found that full-shift airborne fiber concentrations were within or well within the current OSHA 8-hour PEL of 0.1 f/cc [30, 43, 44].

This study evaluated several scenarios that were not previously addressed in the published literature, including the following: (1) the operation of a crane with asbestos-containing brakes and clutches adjacent to the operator inside the cab (Figure 1(e)), and (2) separate analyses of the cleaning of heavy equipment friction linings with an electric wire brush, the hand sanding of linings with compressed air cleaning, and the isolated evaluation of compressed air blowout of linings (Figure 1 and Table 3). Airborne chrysotile fiber concentrations during these specific activities and over the full 8-hour work shift resulted in airborne concentrations below both the 30-minute and full-shift PELs for asbestos from OSHA of 1 f/cc and 0.1 f/cc, respectively. The mechanic during this study also performed a nonstandard task involving the pneumatic sanding of the entire surface of a used clutch band, lasting more than 3 minutes and yielding a 30-minute TWA concentration of just over 1 f/cc and a 30-minute area concentration at 1.5 m of 0.5 f/cc (PCME). However, the mechanic stated that this was a task he would never perform, and it was therefore not representative of the maintenance tasks required and was not included in the study results or tables. Furthermore, the full-shift airborne chrysotile concentrations during this day averaged 0.0414 f/cc (PCME), which indicated that this nonstandard activity did not result in airborne concentrations exceeding the 8-hour OSHA PEL.

With respect to exposure potential associated with activities that have been previously analyzed and reported, including heavy equipment maintenance work, compressed air blowout, sweeping/cleanup, and the handling and shakeout of clothing worn during maintenance tasks, the results from the current study were consistent with other published studies in the peer-reviewed literature, which also found that full-shift TWA airborne fiber concentrations, when reported, were below the current 8-hour OSHA PEL of 0.1 f/cc [38, 41, 55, 66, 73]. For specific activities related to heavy equipment maintenance work, Boelter et al. [41] reported full-shift personal airborne asbestos concentrations averaging 0.014 f/cc PCME (range 0.002 to 0.041 f/cc) and area airborne asbestos concentrations with a mean of 0.011 f/cc PCME (range 0.005–0.022 f/cc). Madl et al. [55] provided an analysis of short-term (30-minute) airborne asbestos concentrations during the disassembly and removal of brakes and reported personal airborne fiber concentrations of 0.024 f/cc PCME (range 0.001–0.09 f/cc). During the operation of heavy equipment, Spencer (2003) found that airborne fiber concentrations were below the LOD and that no asbestos fibers were detected in any of the samples analyzed [72], while in the present study, similarly low concentrations were measured with a single chrysotile fiber detected and an average chrysotile concentration of 0.005 f/cc PCME. Regarding clothes handling, the mean calculated 8-hour TWA airborne chrysotile concentration for the clothes handler comprised approximately 0.2% of the mean full-shift airborne concentration for the mechanic, consistent with previous studies [66, 73].

For the area samples collected in this study, the relationship between the personal samples and area samples collected at 1.5 m away indicated that, when measurable, airborne fiber concentrations were 10 to 60% of the personal concentrations, which is consistent with previous analyses of area samples at similar distances [74]. Furthermore, a comparison of the personal and bystander airborne chrysotile concentrations in this study suggested that the area concentrations beyond 1.5 m, and specifically those collected at 4.6, 9.1, and 9.6 m, did not appear to be influenced by any fiber release associated with the activities at the mechanic source location, given their consistency and similarity with each other. This result suggests it is unlikely that any detectable fibers traveled as far as 4.6, 9.1, or 9.6 m from the source in this study.

A variety of approaches have been proposed for calculating statistics with datasets that include ND samples [75]. Following U.S. EPA guidance [60] for risk assessments involving airborne asbestos measurements, we substituted a value of zero for ND when calculating average airborne concentrations. Alternative approaches including substitution of the detection limit or 1/2 the detection limit would not have impacted the finding in this study that exposures were consistently below the 8-hour TWA OSHA PEL and 30-minute excursion limit. Furthermore, all raw data collected during the study are presented in Tables 2 and 3, or the Discussion section, and therefore, such alternate treatments of the study data points which were below the LOD could be calculated by the reader if desired.

The SEM analysis of airborne fibers collected during the study demonstrated that, similar to previous brake and clutch studies, there was debris attached to airborne chrysotile fibers collected during the study (Figure 6) [9, 55]. Previous research has indicated that the rate of particle removal from the air can be substantially affected by the dimensions and weight of the individual particles. For example, heavier particles such as fibers with attached binder material are likely to be removed from the air more rapidly than lighter particles such as unattached chrysotile fibers, thereby reducing the potential for airborne exposure [76].

The airborne concentration data collected for the chrysotile-containing products used during the brake and clutch work in this study appear to meet the criteria in the exemption language specified by OSHA for labeling of encapsulated materials containing asbestos [12, 59, 77]. In 1972, OSHA first required that “[c]aution labels shall be affixed to all … products containing asbestos fibers, or to their containers, except that no label is required where asbestos fibers have been modified by a bonding agent, coating, binder, or other material so that during any reasonably foreseeable use … no airborne concentrations of asbestos fibers in excess of the exposure limits … will be released” [77]. It was not specified in the U.S. Federal Register who or what party was responsible for this labeling requirement. This exemption still stands today [12].

## 5. Conclusions

The results of this study indicated that airborne chrysotile concentrations during routine friction lining maintenance work on nonautomated crane equipment had a mean range of 0.0053 to 0.0273 f/cc (PCME) over 3.3 to 6.2 hours. Furthermore, full-shift maintenance work on brakes and clutches on this equipment, including bench work such as compressed air use exceeding two minutes per lining, electric wire brush cleaning or hand sanding of chrysotile-containing linings followed by compressed air cleaning, as well as riveting and countersinking of woven brake linings that were not predrilled, collectively resulted in full-shift average airborne chrysotile concentrations of 0.0414 to 0.0445 f/cc (PCME) over 6.4 to 8.5 hours, which was below the current 8-hour TWA OSHA PEL. Personal short-term samples (14–36 minutes) for lining removal, installation, wire brushing, hand sanding, and compressed air use ranged from ND to 0.238 f/cc (PCM and PCME), which was below OSHA's 30-minute excursion limit of 1 f/cc. In addition, personal short-term airborne concentrations during the operation of the crane equipment were between ND and 0.01 f/cc (mean 0.005 f/cc) (PCME), and 30-minute personal samples during clothes handling following crane maintenance work were between ND and 0.0022 f/cc (mean 0.0011 f/cc) (PCME). These data add to the limited information in the literature evaluating the potential for asbestos exposure during the operation and maintenance of nonautomated crane equipment, including data for tasks not previously evaluated. The results are likely to be useful for evaluating asbestos exposure potential during both the historic and present-day use of nonautomated heavy equipment. The data will also be useful for farmers, construction workers, and vehicle maintenance workers who choose to continue to use and maintain such equipment due to its lower cost and simplicity of maintenance in certain scenarios. Overall, the results indicated that full-shift measured airborne chrysotile concentrations during the brake and clutch maintenance activities evaluated here remained below the OSHA 8-hour TWA PEL for asbestos of 0.1 f/cc. For those who continue to use older equipment with chrysotile-containing friction linings, exposures can further be reduced by using wet methods, local exhaust ventilation (LEV), and HEPA vacuums for dust collection and control. Local regulations regarding control measures should always be consulted and followed.

## Figures and Tables

**Figure 1:** Images of study equipment and activities. (a) Bucyrus-Erie 22B crane. (b) Crane and dragline. (c) Using compressed air to blow out rivet holes. (d) Grinding off rivet heads from back side of clutch band to remove linings. (e) Brake and clutch band assembly adjacent to operator seat on 22B. (f) Cleaning used linings with electric wire brush. (g) Sanding used linings with sandpaper. (h) Replacement brake and clutch linings.

**Figure 2:** Diagram of the repair garage. Black dots indicate the main work areas (workbench, 22B crane, and 15B crane). White boxes indicate the area sampling locations and note the distance from each work area.

**Figure 3:** Sequence and approximate durations of maintenance and operation activities over the course of the study. Air sampling durations are noted elsewhere. “Additional Maintenance Tasks” were performed with bands and linings that were removed from the cranes prior to the start of the study. For Tasks #1, 2, and 5, “settling” refers to a period of inactivity during which airborne fibers may settle.

**Figure 4:** Comparison of OSHA's excursion limit (1 f/cc, dashed line) to personal breathing-zone chrysotile concentrations (PCME) for task-based samples with sampling durations of approximately 30 minutes or less (14–36 minutes). Averages (bars) and individual measurements (circles) are represented.

**Figure 5:** Paired personal (gray) and 1.5 m area (black) samples were collected during bench work tasks. Only pairs with sampling durations of approximately 30 minutes or less (11–33 minutes) and with personal samples above the analytical sensitivity limit are shown. The dashed line represents OSHA's excursion limit (1 f/cc).

**Figure 6:** Scanning electron microscope (SEM) image of a debris/fiber cluster collected during the study. The entire length of the scale bar is 10 *μ*m; the filter pore size (visible as black dots) was 0.4 *μ*m.

**Table 1:** Overview of air samples collected during crane maintenance^A^.

Day	Crane maintenance	Additional maintenance tasks^B^	Personal samples	Full-shift area samples (one sample/day)	Number of task-based area samples (1.5 m from workbench, 18–21 m from cranes)^C^
1	Clutch band removed from 22B crane, relined, and almost completely reinstalled; shop cleanup	None	1 full-shift; 2 partial-shift; 5 task-based	1.5 m from 22B crane; 4.6 m from 22B crane; 9.1 m from 22B crane; 4.6 m from workbench; 9.6 m from workbench;	4 samples

2	Finished reinstalling 22B clutch band; brake bands removed from 22B crane, relined, and reinstalled; shop cleanup	(1) Compressed air blowoff of brake linings (2) Compressed air blowoff of clutch linings	1 full-shift; 2 partial-shift; 9 task-based	1.5 m from 22B crane; 4.6 m from 22B crane; 9.1 m from 22B crane; 4.6 m from workbench; 9.6 m from workbench;	9 samples

3	Clutch and brake bands removed from 15B crane, and clutch bands relined; shop cleanup	(3) Sanded brake linings and blew off with compressed air (4) Removed brake linings, cleaned and painted brake bands (5) Cleaned brake lining surface with electric wire brush (6) Measured, cut, and installed woven brake linings	1 full-shift; 2 partial-shift; 8 task-based	1.5 m from 15B crane; 4.6 m from 15B crane; 9.1 m from 15B crane; 4.6 m from workbench; 9.6 m from workbench;	8 samples

^A^Samples were collected in accordance with the NIOSH methods 7400 and 7402. Flow rates were approximately 1-2 L/min for personal samples and 5 L/min for area samples. ^B^Tasks performed on brake and clutch bands that were removed from the crane prior to the start of the study. ^C^Task-based area samples were collected 1.5 m from workbench, including during tasks performed on the cranes which were 18.3 to 21.3 m from the stationary sampler.

**Table 2:** Full-shift and half-shift samples during clutch and brake work.

Sample	Duration (hr)	Volume (L)	PCM—fiber concentration (f/cc)	PCME—chrysotile concentration (f/cc)
Indoor				
Personal—day 1				
Full-shift	6.15	380	0.0136	0.0053
1st half-shift	3.33	391	0.0182	0.0132
1st half-shift	3.30	388	0.0278	0.0225
2nd half-shift	2.75	330	0.0163	0.0077
Average full-shift^A,B^			0.0168	0.0093

Personal—day 2				
Full-shift	8.45	510	<0.0053	—
1st half-shift	3.62	215	<0.0125	—
2nd half-shift	4.78	285	0.1454	0.1454
Average full-shift^A,C^			0.0414	0.0414

Personal—day 3				
Full-shift	6.42	360	0.0368	0.0359
1st half-shift	2.70	161	0.096	0.0960
2nd half-shift	3.67	205	0.0215	0.0215
Average full-shift^A^			0.0449	0.0445
Average full-shift—days 1, 2, and 3			0.0344	0.0317

Area: 1.5 m from crane				
Day 1—crane 22B	6.40	1922	0.0029	0.0012
Day 2—crane 22B	9.02	2696	0.0028	0.0025
Day 3—crane 15B	6.73	2019	0.0030	0.0030
Average full-shift			0.0029	0.0023

Area: 4.6 m from crane				
Day 1—crane 22B	6.28	1907	0.0017	0.0009
Day 2—crane 22B	8.92	2899	0.0035	0.0035
Day 3—crane 15B	7.93	2381	0.0027	0.0027
Average full-shift			0.0026	0.0024

Area: 9.1 m from crane				
Day 1—crane 22B	5.62	1686	0.0019	0.0011
Day 2—crane 22B	8.93	2659	0.0048	0.0047
Day 3—crane 15B	8.28	2474	0.0018	0.0017
Average full-shift			0.0028	0.0025

Area: 4.6 m from workbench				
Day 1	6.07	1850	0.0025	0.0008
Day 2	8.93	2744	0.0029	0.0028
Day 3	8.80	2688	0.0036	0.0036
Average full-shift			0.0030	0.0024

Area: 9.6 m from workbench				
Day 1	5.78	1750	0.0029	0.0016
Day 2	8.98	2744	0.0038	0.0038
Day 3	8.87	2691	0.0032	0.0032
Average full-shift			0.0033	0.0029

Outdoor				
Day 1—full shift	7.33	2380	<0.0011	—
Day 1—full shift	7.33	2197	<0.0012	—
Day 2—partial shift^D^	5.47	1761	<0.0015	—
Day 2—partial shift^D^	3.82	1142	0.0034	0.0034
Day 3—full shift	7.42	2202	<0.0012	—
Day 3—full shift	7.32	2144	<0.0013	—
Average full-shift^C^			0.00047	0.00047

^A^The half-shift samples were averaged (weighted by time) to calculate a second full-shift concentration for each day. The measured and calculated full-shift concentrations were averaged to yield the daily average full-shift concentration. ^B^On day 1, there were two samplers consecutively operating for the duration of the first half of the shift. These two samples were averaged together before the calculations described in footnote (a) were carried out. ^C^To calculate an average concentration, PCM measurements below the analytical sensitivity were assigned a value of zero. Likewise, the corresponding chrysotile-specific concentrations (PCME) were assumed to be zero. ^D^ On day 2, outdoor sampling was conducted at a single location. The sampling stand blew over part way through the day, at which time the sampler was replaced. The full-shift TWA concentration for day 2 is 0.0014 f/cc (PCME).

**Table 3:** Personal and area task-based samples during brake and clutch work, crane operation, and clothes handling. Brake and clutch repair tasks are listed in the order they were performed.

Activity	Tasks	Sample type	Duration (min)	Volume (L)	PCM—fiber concentration (f/cc)	PCME—chrysotile concentration (f/cc)
Clutch and brake work—day 1						
Crane 22B- clutch replacement	Removed clutch band from crane (loosened rusted bolts with pneumatic impact tool)	Personal^A^	200	391	0.018	0.013
			198	388	0.028	0.022
Crane 22B- clutch replacement	Removed clutch band linings at workbench (removed rivets with electric grinder, punch, and hammer); cleaned clutch band surface with electric wire brush; blew off debris with compressed air; painted metal band; cut bulk samples from 2 linings	Personal	38	76	0.077	0.036
		Area (1.5 m)	35	180	<0.015	—
Crane 22B- clutch replacement	Installed new linings on clutch band using rivets at workbench	Personal	36	72	<0.0375	—
		Area (1.5 m)	41	211	<0.0128	—
Crane 22B- clutch replacement	Began installing clutch band with new linings on crane	Personal	72	143	<0.0189	—
		Area^B^ (21.3 m)	113	580	<0.0047	—
Cleanup	Swept up debris from work bench, 22B crane, and floor around the workbench and crane	Personal	30	60	<0.0450	—
		Area^B^ (21.3 m)	113	580	<0.0047	—

Clutch and brake work—day 2						
Crane 22B- clutch and brake work	Finished installing clutch band and then removed brake bands from crane (tightened bolts with pneumatic impact tool)	Personal	151	301	0.032	0.029
		Area (21.3 m)	97^C^	492	<0.0055	—
Crane 22B-brake replacement	Removed brake band linings at workbench (removed rivets with electric grinder, punch, and hammer)	Personal	31	62	0.059	0.041
		Area (1.5 m)	32	156	<0.0173	—
Crane 22B- brake replacement	Cleaned brake band surfaces by pneumatic sanding at workbench; blew off debris with compressed air; painted metal bands	Personal	28	56	<0.0482	—
		Area (1.5 m)	27	139	<0.0194	—
Crane 22B- brake replacement	Installed new linings on brake bands using rivets at workbench	Personal	31	62	<0.0435	—
		Area (1.5 m)	26	123	<0.0219	—
Crane 22B- brake replacement	Continued installing new linings on brake bands using rivets at workbench	Personal	25	50	<0.0539	—
		Area (1.5 m)	31	161	<0.0168	—
Crane 22B- brake replacement	Installed brake bands with new linings on crane	Personal	98	195	0.050	0.044
		Area (21.3 m)	42^D^	203	<0.0133	—
Additional maintenance tasks at workbench^E^	Task #1: blew off a set of used 22B brake linings (1 min 19 sec) and a set of used 15B brake linings (38 sec) that were still on their bands with compressed air	Personal	31	62	0.186	0.186
		Area (1.5 m)	31	150	0.085	0.085
Additional maintenance tasks at workbench^E^	Task #2: blew off used 22B clutch linings that were previously sanded with pneumatic sander (1 min 22 sec) and a set of used 15B clutch linings (53 sec) that were still on their bands with compressed air	Personal	29	57	0.155	0.141
		Area (1.5 m)	30	156	0.087	0.082
Cleanup	Swept up debris from work bench, 22B crane, and floor around the workbench and crane	Personal	31	62	0.059	0.000
		Area (1.5, 21.3 m)^F^	33	159	0.051	0.051
Clutch and brake work—day 3						
Additional maintenance tasks at workbench^E^	Task #3: ground off rivet heads on a set of 22B brake bands with electric grinder; hand-sanded the linings while still on their bands (about 4 min); blew off debris with compressed air (about 1 min)	Personal	32	64	0.238	0.238
		Area (1.5 m)	27	136	0.022	0.018
Additional maintenance tasks at workbench^E^	Task #4: removed rivets on 22B brake bands with punch and hammer; removed linings; cleaned brake bands using electric wire brush; blew off debris with compressed air; painted metal brake bands	Personal	14	28	0.140	0.140
		Area (1.5 m)	11	58	<0.0465	—
Additional maintenance tasks at workbench^E^	Task #5: cleaned a set of used 22B brake linings that were still on their bands with electric wire brush (about 2 min)	Personal	30	60	0.204	0.189
		Area (1.5 m)	30	158	0.037	0.037
Additional maintenance tasks at workbench^E^	Task #6: installed woven brake linings on 22B brake band-cut lining to length with hacksaw (about 15 sec); used pneumatic drill to make approximately 30 rivet holes and countersink linings; blew debris from holes with compressed air; attached woven linings to brake band with rivets.	Personal	60	118	0.260	0.260
		Area (1.5 m)	61	320	0.040	0.040
Crane 15B- brake and clutch work	Removed brake and clutch bands from crane	Personal	108^G^	216	0.024	0.020
		Area (18.3 m)	129	680	0.007	0.003
Crane 15B- clutch work	Removed linings from clutch band at workbench (removed rivets with punch and hammer); cleaned clutch band surface with pneumatic sander; blew off debris with compressed air; painted metal band.	Personal	45	87	<0.031	—
		Area (1.5 m)	43	223	<0.0121	—
Crane 15B- clutch work	Installed new linings on clutch band at workbench (used pneumatic drill to widen about 50 holes in lining and band to fit existing rivets)	Personal	44	87	0.048	0.039
		Area (1.5 m)	43	222	<0.0122	—
Cleanup	Swept up debris from work bench, 15B crane, and floor around the workbench and crane^H^	Area (1.5, 18.3 m)^F^	31	159	<0.017	—

Crane operation—day 3						
Crane operation	Crane operation including swiveling crane and boom, raising and lowering bucket, and scooping motions with bucket (30 min active operation, with engine idle the remaining time)	Personal (L&R lapels)	36	142	0.021	0.010
			34	135	<0.02	—
		Area (2.4 m)	35	140	<0.0193	—
		Area (2.9 m)	38	152	<0.0177	—

Clothes-handling—day 3						
Clothes handling	Handling and shake-out of the three sets of coveralls worn by the mechanic during brake and clutch work on the cranes; approximately the last 2 minutes comprised sweeping up	Personal (L&R lapels)	15	150	0.095	0.000
			15	150	0.079	0.0044
After clothes handling	Samples collected at breathing zone height where the laundry handler was standing; sampling occurred immediately following clothes handling	Area (same location where clothes handler was standing)	15	154	<0.0175	—
			15	154	<0.0175	—

^A^These two samples were also reported on Table 2 since the task duration spanned approximately half the shift. Both samples were collected on the right lapel of the mechanic. No area samples were collected 1.5 m from the workbench during this task. ^B^This area sample spanned the last two consecutive tasks performed on day 1, and thus the results for this sample are listed twice. The area sampler was approximately 21.3 m from the 22B crane and 1.5 m from the workbench. Except for a few minutes spent cleaning the workbench, the mechanic was working at the crane. ^C^This area sample was started 57 minutes after the personal sample. ^D^This area sample was stopped 52 minutes before the personal sample. ^E^The activity “Additional Maintenance Tasks at Bench” refers to work performed at the workbench with brake and clutch linings that were already removed from cranes before the study started. ^F^When the mechanic was cleaning up at the bench, he was approximately 1.5 m from the area sampler, whereas when he was cleaning up at the 22B or 15B crane he was approximately 21.3 or 18.3 m, respectively, from the area sampler. ^G^This personal sample was started 21 minutes after the area sample. ^H^A personal sample was also collected for this task, but the sampling pump shut off prior to the completion of the sampling period, thus the concentration is uncertain.

## Data Availability

All airborne fiber concentrations that resulted from measurements performed have been reported in the study for transparency. The results of individual bulk samples are available upon request. The authors welcome any questions regarding the data collected.
